The article "Effects of cyclooxygenase-2 gene silencing on the biological behavior of SKOV3 ovarian cancer cells" was retracted in 2021. Reasons: duplicated images; duplicated data.

# Effects of cyclooxygenase-2 gene silencing on the biological behavior of SKOV3 ovarian cancer cells

**DOI:** 10.3892/mmr.2014.2732

**Published:** 2014-10-21

**Authors:** FENG-JUN GUO, JING-YAN TIAN, YUE-MEI JIN, LING WANG, RUI-QI YANG, MAN-HUA CUI

**Affiliations:** 1 Department of Obstetrics and Gynaecology, The Second Hospital, Jilin University, Changchun 130041, P.R. China; 2 Department of Urology, Second Division of the First Hospital, Jilin University, Changchun 130021, P.R. China

**Keywords:** ovarian cancer, cyclooxygenase-2, RNA interference, proliferation, invasion, gene therapy

## Abstract

The aim of the present study was to investigate the effects of plasmid-mediated RNA interference targeting of cyclooxygenase-2 (COX-2) on the biological behaviors of SKOV3 human ovarian cancer cells and to analyze the function of COX-2 in carcinogenesis and development of ovarian cancer. A COX-2 small hairpin (sh)RNA sequence was designed and synthesized and pGPU6-COX-2-shRNA plasmids were constructed. The recombinant vector plasmids were stably transfected into SKOV3 cells. The mRNA and protein expression of COX-2 was subsequently analyzed by quantitative polymerase chain reaction and western blot analysis, respectively. MTT and colony formation assays were used to detect the cellular proliferation ability and flow cytometry was performed to detect phase changes in the cell cycle. Finally, a Transwell assay was used to detect cell invasion. The SKOV3 cells, transfected with recombinant vector plasmids, and control cells, were injected into nude mice and the tumor emergence time, volume and weight were measured. The impact of COX-2 gene silencing on the growth of xenograft tumors in nude mice was analyzed. Following transfection of the pGPU6-COX-2-shRNA plasmid, *in vitro* analyses indicated that the shRNA efficiently suppressed the mRNA and protein expression of COX-2. COX-2 gene silencing significantly inhibited the proliferation and invasion ability of SKOV3 cells, leading to cell cycle arrest in G1. The tumor formation time in the interference group was significantly prolonged, and the tumor volume and weight were significantly decreased, as compared with the control group. Plasmid-mediated shRNA was shown to effectively silence COX-2 expression in SKOV3 ovarian cancer cells. It was identified that COX-2 functioned in regulating proliferation, cell cycle and invasion of ovarian cancer cells. These findings provided a theoretical basis for determining the function of COX-2 in the development of ovarian cancer and suggested that COX-2 may be an effective target for gene therapy and clinical applications.

## Introduction

Ovarian cancer is the predominant gynecological malignant tumor that poses a serious and under-recognized threat to the health of females. Ovarian cancer is insidious, and advances gradually, therefore resulting in a low five-year survival rate (1,2). Ovarian cancer has a higher mortality rate in females than all other gynecological cancers combined; therefore, development of novel treatments is required. Cyclooxygenase-2 (COX-2) is an inducible enzyme that is either lowly expressed or absent in normal cells. Under certain conditions, including inflammation, tumors and other pathological conditions, COX-2 is highly expressed, which is associated with upregulation of prostaglandins. Recent studies have identified that COX-2 is closely associated with the development of various types of cancer (3–7). Currently available evidence indicates that COX-2 expression is significantly higher in ovarian cancer tissues compared with benign tumors (8–11). High expression of COX-2 in ovarian cancer tissues is associated with poorer prognosis, shorter survival time and decreased sensitivity to treatment. This suggests that COX-2 may act as an oncogene involved in the development of ovarian cancer. However, the precise role of COX-2 in the development and progression of ovarian cancer, as well as the molecular mechanisms involved in these processes, remain to be elucidated. The present study employed small hairpin (sh)RNA interference technology to observe the effects of COX-2 gene silencing *in vitro* and *in vivo* on the biological behavior of SKOV3 human ovarian cancer cells, to explore the role of COX-2 gene in ovarian cancer development. The present study provided a theoretical basis for COX-2-targeted therapy of ovarian cancer.

The article "Effects of cyclooxygenase-2 gene silencing on the biological behavior of SKOV3 ovarian cancer cells" was retracted in 2021. Reasons: duplicated images; duplicated data.

## Materials and methods

### Cell lines and experimental animals

The SKOV3 human ovarian cancer cell line and *E. coli* DH5 alpha strain were purchased from the Shanghai Biological Cell Bank, Chinese Academy of Sciences (Shanghai, China). Female SPF BALB/C nude mice (n=18) (4–5 weeks of age; 17–20 g body weight) were purchased from the Shanghai Slack Laboratory Animal Center (Shanghai, China). The mice were housed in a temperature-controlled and closed aseptic environment (at a constant temperature of 18–22°C and humidity of 50–80%) under a 12-h light/dark cycle, and provided free access to sterile water and food. The experiments were carried out according to the guidelines and practices established by the ethics committee of The Second Hospital, Jilin University (Changchun, China).

### Plasmids

Plasmid pGPU6/GFP/Neo was purchased from Shanghai GenePharma Co., Ltd. (Shanghai, China).

### Primer sequences

The following primers were used: COX-2 upstream, 5′-TCAAGTCCCTGAGCATCTAC-3′ and downstream, 5′-CATTCCTACCACCAGCAACC-3′; GAPDH upstream, 5′-GCACCGTCAAGGCTGAGAAC-3′ and downstream, 5′-TGGTGAAGACGCCAGTGGA-3′. The primers were synthesized by Dalian Takara Bio Company Limited (Shiga, Japan).

The article "Effects of cyclooxygenase-2 gene silencing on the biological behavior of SKOV3 ovarian cancer cells" was retracted in 2021. Reasons: duplicated images; duplicated data.

### Selection of COX-2 RNA target sequence, shRNA design and synthesis

Human COX-2 siRNA target sequence was designed according to literature searches (12) as follows: 5′-GGACTTATGGGTAATGTTA-3′. Considering the *Bbs*I and *Bam*HI restriction sites in the plasmid, ‘CACC’ was added to the 5′ cohesive end on the sense strand and ‘GATC’ was added to the 5′ cohesive end on the antisense strand. ‘TTTTTT’ was added as the transcription termination sequence. A ‘G’ nucleotide was inserted into the plasmid in order to preserve the *Bam*HI restriction site. The LOOP structure was designed as TTCAAGAGA. The final COX-2 shRNA sequence was designed as follows: sense, 5′-CACCGGACTTATGGGTAATGTTATTCAAGAGATAACATTACCCATAAGTCCTTTTTTG-3′ and antisense, 5′-GATCCAAAAAAGGACTTATGGGTAATGTTATCTCTTGAATAACATTACCCATAAGTCC-3′. COX-2 shRNA was synthesized by Shanghai Gemma Bio-tech, Inc.

### Reagents

A quantitative polymerase chain reaction (qPCR) kit was purchased from Takara. A Total RNA Extraction TRIzol™ Reagent kit was from Fermentas (Pittsburgh, PA, USA); Lipofectamine 2000 was purchased from Invitrogen (Invitrogen Life Technologies, Carlsbad, CA, USA); G418 was from Shanghai PuFei Co.; MTT Kit was purchased from Sigma (Sigma, St Louis, MO, USA); Propidium iodide was purchased from Nanjing Keygen Biotechnology Company; Cell invasion Chamber was obtained from Corning (Corning Inc., Corning, NY, USA).

### Cell culture and transfection

SKOV-3 cells were maintained as monolayer cultures in Dulbecco’s modified Eagle’s medium supplemented with 10% fetal bovine serum and 1% antibiotics in a humidified chamber with 5% CO_2_ at 37°C. COX-2 shRNA double-stranded template was inserted into the pGPU6/GFP/Neo plasmid using an annealing and digestion technique, and the recombinant plasmid pGPU6-COX-2-shRNA was constructed. The plasmid was transformed into *Escherichia coli* competent cells and the positive recombinant colonies were selected and amplified. The extracted recombinant plasmids were digested and subjected to DNA sequencing. The recombinant plasmids were transiently transfected into SKOV3 cells using the Lipofectamine™ 2000 Transfection kit, according to manufacturer’s instructions. Following selection with medium containing G418 for neomycin selection, the resistant clones that stably expressed human COX-2 shRNA were obtained. The resistant clones were gradually amplified followed by routine culture and sub-culture. Following transfection, the fluorescence expression levels were observed under an inverted fluorescence microscope. The experimental groups of plasmid transfection were established as follows: i) Control group (CON), normal SKOV3 cells without plasmid transfection; ii) negative control group (NC), SKOV3 cells transfected with the recombinant negative control plasmid; iii) interference group (KD), SKOV3 cells transfected with pGPU6-COX-2-shRNA recombinant plasmid.

The article "Effects of cyclooxygenase-2 gene silencing on the biological behavior of SKOV3 ovarian cancer cells" was retracted in 2021. Reasons: duplicated images; duplicated data.

### Analysis of COX-2 mRNA expression by qPCR

Following stable transfection, total RNA was isolated with TRIzol^®^ reagent according to the manufacturer’s instructions. The qPCR cycling conditions were 95°C for 5 min; 94°C for 30 sec, 55°C for 30 sec, 72°C for 30 sec, for 30 cycles; 72°C for 10 min; 4°C for 5 min. COX-2 mRNA content was analyzed using a gel image analysis system (BioCapMW software 11.01; Microsoft, Redmond, USA).

### Western blot analysis

COX-2 protein expression was analyzed by western blotting. Briefly, total cellular protein (30–50 μg) was subjected to 7.5% SDS-PAGE and electrotransferred onto a polyvinylidene fluoride membrane (Bio-Rad, Hercules, CA, USA). Following blocking with 5% nonfat dry milk in 10 mM Tris, pH 7.5, containing 0.15 M NaCl and 0.05% Triton X-100, the membranes were probed with a mouse monoclonal anti-COX-2 antibody (1:500 in 5% milk; Cayman Chemical, USA). The membranes were then washed and incubated with horseradish-peroxidase conjugated secondary antibody (goat anti-mouse; 1:2000 in 5% milk; Bio-Rad). Protein bands were visualized using a chemiluminescent detection system. The relative expression of COX-2 protein was analyzed using Quantity One v.4.62 software (Bio-Rad).

### MTT assay

The proliferation status of SKOV3 cells was determined by MTT assay. SKOV3 cells were seeded at a density of 1×10^4^ cells per well in a flat-bottomed 96-well microplate. The cells were incubated in 5% CO_2_ at 37°C for 12 h. After 1, 2, 3, or 4 days incubation, 10 μl MTT was added to each well and further incubated for 4 h. The supernatant was then removed and 100 μl dimethyl sulfoxide was added. It was agitated for 10 min until the crystals dissolved. The optical density (OD) at 490 nm was measured using an ELISA reader (Molecular Devices Corp, Sunnyvale, CA, USA). The negative control well contained no cells, and its OD was subtracted from that of the other samples. Each well was read three times in triplicate.

### Colony forming assay

SKOV cells were seeded in triplicate at 1,000 cells/well in six-well plates in complete medium. After 2–3 weeks of growth in 5% CO_2_ at 37°C, the cells were fixed with 5 ml paraformaldehyde for 15 min and stained with the appropriate amount of Giemsa staining solution for 15 min, and the grossly visible colonies were counted. All experiments were repeated at least three times. Groups that consisted of >50 cells were counted as a clone. The plating efficiency was determined as the number of colonies formed divided by the total number of cells plated.

The article "Effects of cyclooxygenase-2 gene silencing on the biological behavior of SKOV3 ovarian cancer cells" was retracted in 2021. Reasons: duplicated images; duplicated data.

### Cell cycle analysis by flow cytometry

The total number of cells collected was >10^4^. Propidium iodide (PI) was added to the cells, which were analyzed by flow cytometry (EPICS XL; Beckman Coulter, Miami, FL, USA). The proliferation index was calculated using the following formula: Proliferation index = (S + G2/M) / (G0/G1 + S + G2/M).

### Transwell cell culture chamber assay

An invasion assay was employed to assess the ability of SKOV3 cells to invade a synthetic basement membrane. Transwell chambers (Corning, Inc.) with a polycarbonate filter (6.5-mm pore size), separating the upper and lower chambers, were used. SKOV3 cells in the exponential growth phase were digested using trypsin, and a single cell suspension was prepared. The cell density was adjusted to 2.5×10^6^/ml. The assay was performed in accordance with the Transwell Chamber instructions of Corning Company. The non-invading cells on the top surface of the filter membrane were removed using a cotton swab. Cells on the bottom surface of the filter were counted, and the mean number of cells was determined from five high-power fields under a light microscope (Olympus FP50; Olympus Tokyo, Japan). Each experiment was performed three times in triplicate.

### Xenograft model

Eighteen nude mice were randomly divided into three groups (six mice/group), which were marked as CON, NC and KD, respectively. The three groups of nude mice were inoculated with SKOV3 cells, SKOV3 cells transfected with negative control recombinant plasmid and SKOV3 cells transfected with pGPU6-COX-2-shRNA recombinant plasmid, respectively. Each group of nude mice was transferred to a clean bench and underwent strong iodine disinfection. The cell suspension (0.2 ml, ~5×10^7^ cells) was subcutaneously injected into the left armpit of BALB/C nude mice using a 1-ml syringe. Following inoculation, the nude mice were maintained in a pathogen-free sterile environment with appropriate temperature and free access to sterile water and food. Following inoculation with different SKOV3 cells as indicated, the subcutaneous tumor growth in nude mice was observed daily. The tumor inoculation time and the survival conditions of the nude mice bearing a tumor were recorded. Tumors exceeding 3 mm in diameter were recorded as positive (tumorigenic standard). Following tumor development, the long and short radius of the implanted tumors was measured every seven days. In addition, the volume of the tumor was calculated (volume = 1/2 long radius × short radius^2^). Following 28 days of tumor development, the nude mice were sacrificed by cervical vertebrae dislocation. The tumors were separated, the tumor volume and weight were measured, and images of the tumors were captured (Olympus E-M10; Olympus, Tokyo, Japan). The tumor inhibition rate was calculated using the following formula: Tumor inhibition rate = (tumor weight of control group - tumor weight of experimental group)/tumor weight of control group ×100%.

The article "Effects of cyclooxygenase-2 gene silencing on the biological behavior of SKOV3 ovarian cancer cells" was retracted in 2021. Reasons: duplicated images; duplicated data.

### Statistical analysis

All statistical analyses were performed using SPSS 13.0 software (SPSS, Chicago, IL, USA). Values are expressed as the mean ± standard deviation. Statistical comparisons were performed using an independent Student’s t-test and one-way analysis of variance. P<0.05 was considered to indicate a statistically significant difference between values.

## Results

### Identification of PGPU6-COX-2-shRNA recombinant plasmid by DNA sequencing

The positive recombinant plasmids were identified by Shanghai Yingjun Biotechnology Co., Ltd. (Shanghai, China). The obtained sequence was compared to the previously synthesized sequence. As indicated in Fig. 1, the sequencing results confirmed that the pGPU6-COX-2-shRNA recombinant plasmid matched the expected DNA sequences and the COX-2 shRNA sequence was inserted correctly, suggesting a successful construction of recombinant plasmid.

### Stable transfection of SKOV3 cells with recombinant plasmid

Following antibiotic selection with G418, SKOV3 cells that stably expressed the recombinant plasmid were obtained. Fluorescence microscopy identified that the majority of SKOV3 cells expressed green fluorescent protein for different lengths of time (10, 20, 30 and 40 d). Comparison with the transmitted light images showed that the transfection efficiency of the different groups was >90%, which was suitable for the subsequent experiments (Fig. 2).

### Confirmation of COX-2 silencing

SKOV3 cells were transfected with pGPU6-COX-2-shRNA and recombinant negative control plasmid, respectively. Total RNA was extracted and COX-2 mRNA was detected by qPCR. As shown in Fig. 3, as compared with the CON and NC cells, COX-2 mRNA expression levels in the KD cell group were significantly decreased (P<0.05). There was no statistically significant difference in the mRNA expression levels between the CON and NC groups (P>0.05). Furthermore, the total protein was extracted from the SKOV3 cells and levels of COX-2 were detected by western blot analysis. As shown in Fig. 4, as compared with the CON and NC cells, the COX-2 protein expression levels in the KD cell group were significantly decreased (P<0.05). There was no statistically significant difference in protein expression levels between CON and NC groups (P>0.05).

The article "Effects of cyclooxygenase-2 gene silencing on the biological behavior of SKOV3 ovarian cancer cells" was retracted in 2021. Reasons: duplicated images; duplicated data.

### COX-2 gene silencing reduces SKOV3 cellular proliferation

The MTT method was used to assess the cellular proliferation ability following COX-2 gene silencing. As indicated in Fig. 5, as compared with the CON and NC groups, the number of live cells in the KD group was significantly decreased, suggesting that following the inhibition of COX-2 expression, SKOV3 cellular proliferation ability and growth were significantly reduced. The cell proliferation ability in the KD group following 24 h showed significant differences as compared with the NC and CON groups (P<0.05). There was no statistically significant difference in the cell proliferation ability between the CON and NC groups (P>0.05).

### COX-2 gene silencing reduces colony formation ability of SKOV3 cells

As indicated in Fig. 6, the colony size in the KD group was significantly reduced as compared with the CON and NC groups. The colony-forming number in the KD group was 131±14, whereas that of the CON and NC groups was 240±20 and 210±30, respectively. The number of colonies in the KD group was significantly reduced as compared with that in the CON and NC groups (P<0.05). There was no statistically significant difference between the CON and NC groups (P>0.05).

### COX-2 gene silencing causes G1 phase arrest and reduces the proliferative index of SKOV3 cells

The effect of COX-2 gene silencing on the SKOV3 cell cycle was detected PI staining and flow cytometric quantification. As indicated in Table I, compared with the CON and NC groups, the number of cells in G1 phase in the KD group was considerably increased and the cell number in S and G2 phase was significantly reduced (P<0.05). There was no statistically significant difference in the cell cycle distribution between the CON and NC groups (P>0.05). The proliferation index in the KD group was significantly lower than that in the CON and NC groups. The apoptotic peak was not identified in all three groups.

### COX-2 gene silencing attenuates SKOV3 cell invasiveness

In the Transwell assay, the number of cells penetrating the membrane in the CON, NC and KD groups was 85±9, 79±7 and 38±5, respectively. The number of cells penetrating the membrane in the KD group was significantly reduced as compared with that in the NC and CON groups (P<0.05). There was no statistically significant difference between the CON and NC groups (P>0.05) (Fig. 7). These results suggested that inhibition of COX-2 expression significantly attenuated SKOV3 cell invasiveness.

### Establishment of a SKOV3 xenograft model

In the present study, the success rate of subcutaneous implantation tumors in 18 nude mice was 100%. During the experiment, the growth conditions of the tumor-bearing nude mice and their diets were normal. There were no mortalities or abnormal behavior. The tumors appeared ~7 days following inoculation of the cells in the CON and NC groups, and 10 days following inoculation in the KD group.

The article "Effects of cyclooxygenase-2 gene silencing on the biological behavior of SKOV3 ovarian cancer cells" was retracted in 2021. Reasons: duplicated images; duplicated data.

### Effects of COX-2 gene silencing on the growth of SKOV3 xenograft tumors in nude mice

From day 7 of inoculation, the long and short radius of the xenograft tumors in tumor-bearing nude mice was measured every seven days, and the volume of the tumor was calculated. As indicated in Table II, the tumor volume in the KD group was significantly lower as compared with that in the CON and NC groups (P<0.05). There was no statistically significant difference between the CON and NC groups. Twenty-eight days following tumor development, the nude mice were sacrificed by cervical dislocation and the tumors were extracted. The pink tumors presented round or oval-shaped and had a complete capsule, medium texture and a clear boundary (Fig. 8). The average tumor weight in the KD group was significantly lower as compared with the CON and NC groups (P<0.05). When compared with the blank control group, the tumor inhibition rate was 41.45%. As compared with the negative control group, the tumor inhibition rate was 43.62%. There was no statistically significant difference between the CON and NC groups.

## Discussion

In the present study, a COX-2 shRNA sequence was designed and synthesized according to the COX-2 gene sequence, and a pGPU6-COX-2-shRNA recombinant plasmid vector was constructed. The recombinant plasmid pGPU6-COX-2-shRNA was transiently transfected into SKOV3 cells. In addition, it was shown through *in vitro* and *in vivo* experiments that COX-2 expression may have an important role in the proliferation, growth, invasion and metastasis of ovarian cancer cells.

The results of the MTT and colony formation assays demonstrated that COX-2 gene silencing significantly inhibited the proliferation and viability of ovarian cancer cells, suggesting that COX-2 promoted the proliferation and viability of ovarian cancer cells.

Cells that are growing and dividing go through a repeated series of events leading to division and duplication (replication), known as the cell cycle or cell-division cycle. In this process, the genetic material of the cells is copied and equally distributed to both daughter cells. As the cellular DNA content in each period of the cell cycle is different, using the DNA-binding dye, propidium iodide (PI), the cell cycle and cell proliferation was detected using a flow cytometer. The results of the present study demonstrated that following COX-2 gene silencing in SKOV3 cells, the cell cycle was blocked in G1 phase and the number of cells in the DNA synthesis phase was significantly reduced, resulting in reduced DNA synthesis as well as cell proliferation inhibition. This data implies that COX-2 promoted tumor cell proliferation through modulation of the cell cycle. The mechanism by which COX-2 regulates cell cycle progression still requires further in-depth studies.

The article "Effects of cyclooxygenase-2 gene silencing on the biological behavior of SKOV3 ovarian cancer cells" was retracted in 2021. Reasons: duplicated images; duplicated data.

Among the invasive and metastatic processes of malignant tumors, the critical step is to degrade the extracellular matrix (ECM) and basement membrane and break the natural barrier, thus allowing for tumor cell spread (13). The Transwell invasion assay is a commonly used test for the effective analysis of the cell invasion ability. The results of the present study suggested that COX-2 gene silencing decreased the number of cells penetrating the membrane and therefore inhibited the invasion ability of SKOV3 cells, implying that COX-2 promoted the invasion ability of ovarian cancer cells and was conducive to the spread and metastasis of ovarian cancer. The possible underlying mechanism involves matrix metalloproteinases (MMPs), vascular endothelial growth factor (VEGF) and other cytokines (14). MMPs are Ca^2+^- and Zn^2+^-dependent endopeptidases that function in the degradation of various ECM components (13). MMPs are enzymes implicated in normal and pathological tissue remodeling processes, wound healing, angiogenesis and tumor invasion (13–15). Using immunohistochemical technology, previous research has detected COX-2, MMP-9 and VEGF expression in epithelial ovarian cancer, borderline ovarian tumors and normal ovarian tissue (16). It was shown that COX-2 protein expression was positively correlated with expression of MMP-9 and VEGF in epithelial ovarian cancer. It is speculated that COX-2 affects tumor invasiveness through MMP-9 and VEGF. Symowicz *et al* (17) suggested that COX-2 inhibitors may reduce the expression and activity of MMP-2 precursors in ovarian cancer cells. Furthermore, Leung *et al* (18) and Pan *et al* (19) confirmed that COX-2 inhibitors reduced the expression of MMP-2 in colorectal cancer and lung cancer cells.

The present study showed that COX-2 gene silencing decreased tumor development in nude mice and that the tumor volume and weight were significantly lower than those of the blank and negative control groups, indicating that the inhibition of COX-2 gene expression suppressed the growth of ovarian cancer. Therefore, COX-2 may be used as an effective target of gene therapy for ovarian cancer. Lowering the target gene expression *in vivo* is likely to inhibit the growth of ovarian cancer cells, achieving successful ovarian cancer treatment.

The article "Effects of cyclooxygenase-2 gene silencing on the biological behavior of SKOV3 ovarian cancer cells" was retracted in 2021. Reasons: duplicated images; duplicated data.

RNAi technology has been successfully used to silence the COX-2 protein in different *in vitro* and *in vivo* models. Previous investigation demonstrated that the silencing of COX-2 mediated by LV-COX-2-siRNA significantly inhibited growth and induced cell cycle arrest in non-squamous cell lung carcinoma cell lines. In addition, the decreased expression of COX-2 modulated the expression of cell cycle-regulatory genes, up-regulated p21 and down-regulated cyclin D1 (22). The gene knock down of COX-2 in human osteosarcoma cells significantly inhibits the growth and decreases the migration ability of SaOS_2_ cells. Furthermore, it also reduces VEGF, EGF and basic fibroblast growth factor mRNA and protein expression (23). COX-2 siRNA treatment also inhibits cell proliferation and induces apoptosis in esophageal squamous carcinoma EC109 cells (24).

In conclusion, the present study effectively silenced COX-2 gene expression in SKOV3 cells by using plasmid vector-mediated RNA interference technology. In addition, *in vitro* and *in vivo* studies demonstrated that COX-2 gene silencing had important implications in proliferation, cell cycle, colony formation and invasion of ovarian cancer cells. These findings provided a theoretical basis on understanding the role of COX-2 in the development of ovarian cancer and additionally show that COX-2 may be an effective target for gene therapy, which has prospects in clinical applications.

## Figures and Tables

**Figure 1:** Sequencing chromatogram of the pGPU6-small hairpin RNA-cyclooxygenase-2 recombinant plasmid.

**Figure 2:** Assessment of transfection efficiency in SKOV3 cells transfected with recombinant plasmid (magnification, ×20). (A1 and 2) Fluorescent and transmitted light images of SKOV3 cells transfected with pGPU6-cyclooxygenase-2-shRNA recombinant plasmid. (B1 and 2) Fluorescent and transmitted light images of SKOV3 cells transfected with pGPU6-Control-shRNA recombinant plasmid. sh, small hairpin.

**Figure 3:** Cyclooxygenase-2 mRNA expression analysis following quantitative polymerase chain reaction. COX, cyclooxygenase; CON, control; NC, negative control; KD, interference group; bp, base pairs.

**Figure 4:** Western blot analysis of Cyclooxygenase-2 protein expression. COX, cyclooxygenase; kDa, kilodaltons; CON, control; NC, negative control; KD, interference group.

**Figure 5:** Effect of Cyclooxygenase-2 gene silencing on SKOV3 proliferation ability. CON, control; NC, negative control; KD, interference group. Y-axis denotes optical density.

The article "Effects of cyclooxygenase-2 gene silencing on the biological behavior of SKOV3 ovarian cancer cells" was retracted in 2021. Reasons: duplicated images; duplicated data.

**Figure 6:** Result of colony forming experiments. CON, control; NC, negative control; KD, interference group.

**Figure 7:** Cell invasion assay by Transwell method Stained with crystal voolet. (Magnification, ×100). CON, control; NC, negative control; KD, interference group.

**Figure 8:** Analysis of xenograft tumors in nude mice in each group. CON, control; NC, negative control; KD, interference group.

**Table I:** Cell cycle analysis across the experimental groups.

	Cell cycle			
	
Groups	G0/G1 (%)	S (%)	G2/M (%)	Proliferation index (%)
CON	36.34±5.22	30.50±5.12	33.16±2.54	63.66±4.21
NC	37.50±4.54^b^	27.68±4.53^b^	34.82±5.21^b^	62.50±4.63^b^
KD	62.45±5.23^a^	23.53±2.21^a^	14.02±1.93^a^	37.55±3.62^a^

a P<0.05 vs blank control and negative control;

b P>0.05 vs blank control.

Data are presented as the mean ± standard deviation. CON, control; NC, negative control; KD, interference group.

**Table II:** Effect of cyclooxygenase-2 gene silencing on the volume of xenograft tumors.

	Days				
	
Group	7	14	21	28	35
KD	25.2±3.1^a^	37.3±8.1^a^	74.4±10.6^a^	120.9±14.3^a^	204.8±20.8^a^
NC	30.2±4.5^b^	62.7±10.2^b^	128.2±11.5^b^	260.4±21.3^b^	386.5±49.7^b^
CON	31.8±5.2	64.5±13.5	121.3±21.2	271.8±40.2	390.5±45.1

Experiments were performed three times.

a P<0.05 vs blank control and negative control group;

b P>0.05 vs blank control group.

Data are presented as the mean ± standard deviation. Volume unit: mm^3^. CON, control; NC, negative control; KD, interference group.
